# Supplementation with Natural Forms of Vitamin E Augments Antigen-Specific TH1-Type Immune Response to Tetanus Toxoid

**DOI:** 10.1155/2013/782067

**Published:** 2013-07-07

**Authors:** Ammu Kutty Radhakrishnan, Dashayini Mahalingam, Kanga Rani Selvaduray, Kalanithi Nesaretnam

**Affiliations:** ^1^Pathology Division, Faculty of Medicine and Health, International Medical University, 126, Jalan Jalil Perkasa 19, Bukit Jalil, 57000 Kuala Lumpur, Wilayah Persekutuan, Malaysia; ^2^Department of Nutrition, Malaysian Palm Oil Board, 6, Persiaran Institusi, Bandar Baru Bangi, 43000 Kajang, Selangor Darul Ehsan, Malaysia

## Abstract

This study compared the ability of three forms of vitamin E [tocotrienol-rich fraction (TRF), alpha-tocopherol (*α*-T), and delta-tocotrienol (*δ*-T3)] to enhance immune response to tetanus toxoid (TT) immunisation in a mouse model. Twenty BALB/c mice were divided into four groups of five mice each. The mice were fed with the different forms of vitamin E (1 mg) or vehicle daily for two weeks before they were given the TT vaccine [4 Lf] intramuscularly (i.m.). Booster vaccinations were given on days 28 and 42. Serum was collected (days 0, 28, and 56) to quantify anti-TT levels. At autopsy, splenocytes harvested were cultured with TT or mitogens. The production of anti-TT antibodies was augmented (*P* < 0.05) in mice that were fed with *δ*-T3 or TRF compared to controls. The production of IFN-*γ* and IL-4 by splenocytes from the vitamin E treated mice was significantly (*P* < 0.05) higher than that from controls. The IFN-*γ* production was the highest in animals supplemented with *δ*-T3 followed by TRF and finally *α*-T. Production of TNF-*α* was suppressed in the vitamin E treated group compared to vehicle-supplemented controls. Supplementation with *δ*-T3 or TRF can enhance immune response to TT immunisation and production of cytokines that promote cell-mediated (TH1) immune response.

## 1. Introduction

Tocopherol and tocotrienol are bioactive plant derivatives that belong to the vitamin E family. Some of the naturally occurring homologues of tocotrienols are shown in Figure 1. Most of these tocotrienol homologues are found in the palm oil [1]. Tocotrienols are lipid-soluble antioxidants that have been reported to possess many beneficial health benefits that are not usually exhibited by tocopherols [2], such as potent anticancer effects [3], neuroprotective effects [4, 5], and cholesterol lowering properties [6]. To date, there have been some clinical and nonclinical studies highlighting the use of *α*-tocopherols to enhance the immune system in elderly human subjects [7] as well as in aged animals [8–10]. Both tocopherol and tocotrienol supplementation induced immunomodulatory effects resulting in Brown Norway rats [11]. When T-helper cells are appropriately activated, these lymphocytes will differentiate into effector T-cells that secrete distinct types of cytokines. The T-helper-1 (TH1) cells produce cytokines that promote cell-mediated immune responses such as interferon-gamma (IFN-*γ*) whilst the TH2 cells produce cytokines such as IL-4, IL-5 and IL-13, which will activate humoral immune responses [12]. Interferon-*γ* is the signature cytokine for the TH1 immune responses. This cytokine exerts antitumour or antiviral effects by directly inhibiting replication of these cells or by activating the effector cells of the innate immune system such as natural killer (NK) cells, macrophages, and neutrophils [13]. It has been reported that production of IFN-*γ* by T-lymphocytes and NK cells is triggered through the recognition of infected cells or through the involvement of other cytokines [14]. Activated macrophages and dendritic cells secrete IL-12. Interlekin-12 is crucial for activating T-cells to produce IFN-*γ* as well as to provide the signals required for the activation of antigen-specific cytotoxic T-lymphocytes (CTL) [14, 15].

We have previously reported that supplementation of *α*-T or TRF for two months did not produce any significant changes on immune parameters in healthy human subjects in the absence of immunogenic challenge [16]. More recently, we have shown that supplementation of TRF markedly enhanced immune response to tetanus toxoid (TT) vaccine in normal healthy young volunteers [17]. The TRF preparation used in the said study contained 70% tocotrienols and 30% *α*-tocopherol. In the said study, it could not be ascertained which vitamin E isomer contributed to the enhanced immune response observed. Hence, in this study, we used a mouse model, which is similar to our human study to identify the main component in the TRF that could have contributed to the enhanced immune response observed. At the time of this study, we only had the pure forms of the *α*-T and *δ*-T3 available and this was compared with TRF, which was used in the human study [17].

## 2. Materials and Methods

### 2.1. Vitamin E

Tocotrienol-rich fraction (TRF) and *α*-T concentrates were obtained from Golden Hope Plantation, Malaysia. The TRF preparation used contains 70% tocotrienol (113 mg/g *α*-tocotrienol, 91 mg/g *γ*-tocotrienol, 36 mg/g *δ*-tocotrienol, and 10 mg/g *β*-tocotrienol) and 30% tocopherol (78 mg/g *α*-tocopherol and 0.5 mg/g *β*-tocopherol). The *δ*-T_3_ was purchased from Isei, Japan. The purity of each isomer was approximately 97%. The composition of TRF used in this study is *α*-tocopherol (32%), *α*-tocotrienol (25%), *γ*-tocotrienol (29%), and *δ*-tocotrienol (14%). The concentrates of the isomers were then prepared as an emulsion with Soya bean oil to give a final concentration of 20 mg/mL. At the time of this study, only *δ*-T3 was available in the pure form. 

### 2.2. Animals and Experimental Design

Female BALB/c mice (4–6 weeks of age) were purchased from Institute of Medical Research (Kuala Lumpur, Malaysia) and housed in the animal holding facility of the Malaysian Palm Oil Board (Bangi, Malaysia) under stable climatic conditions. Mice were given pellet diet and water *ad libitum*. After one week of adaptation, the mice (*n* = 20) were randomly divided into four groups of five mice each. The mice in each group were orally fed (0.1 mL) with 1 mg of TRF, *α*-T, or *δ*-T3 daily until the mice were sacrificed at the end of the experiment (Figure 2). The mice in the control group were given 0.1 mL of the vehicle, that is, Soya bean oil. All animals were immunised with 4 Lf/mL (0.1 mL) of the alum-adsorbed TT vaccine (Biofarma, Indonesia) on day 14. The TT vaccine was administered intramuscularly in the left hind-leg quadriceps of each mouse. Booster doses of the TT vaccine were given on days 28 and 42 (Figure 2). For all immunisation procedures, the mice were lightly anaesthetised with diethyl ether. Serum samples were obtained via retroorbital bleeding on day 0 (baseline/preimmunisation), day 28 and day 56 (postimmunisation). Sera were stored at −20°C. When the animals were sacrificed on day 56, blood, spleen and adipose tissue were collected for various tests. 

This study was conducted according to the guidelines laid down in the Declaration of Helsinki and all procedures involving human subjects/patients were approved by the Medical Research and Ethics Committee of the International Medical University. Animal care and handling strictly followed the guidelines provided by this committee.

### 2.3. Analysis of Serum Anti-Tetanus Toxoid Antibodies

Serum levels of total anti-TT antibodies were quantified by ELISA. Briefly, 96-well Nunc Maxisorb microtitre plates (Nunc, Gaithersburg, MD) were coated with 100 *μ*L/well of 3 *μ*g/mL of TT solution in 0.05 M sodium carbonate buffer (pH 9.2) overnight at 4°C. Plates were washed using ELISA wash buffer (PBS with 0.05% Tween-20) and blocked with 200 *μ*L/well of ELISA blocking buffer (PBS with 1% (w/v) bovine serum albumin (Fisher Scientific, Pittsburgh, PA)) for two hours at room temperature. Plates were then washed as before. Serum was serially diluted in ELISA blocking buffer and 100 *μ*L of the test samples were added as duplicates to the wells. Serum obtained from nonimmunised animals served as the negative control for this assay. Plates were incubated at room temperature for two hours. After two hours, the plates were washed and 100 *μ*L of appropriately diluted anti-mouse Ig conjugated with horseradish peroxidase (Sigma, St. Louis, MO, USA) was added to all wells. Following a 60 min incubation at 37°C the plates were washed and antibody binding was detected with 100 *μ*L of 3,3′,5,5′-tetramethylbenzidine (TMB) substrate buffer (Sigma, St. Louis, MO). The absorbance was read using an ELISA reader. The anti-TT titres were expressed as the reciprocal of the dilution giving an absorbance value ≤0.45 as described previously [18].

### 2.4. Splenocyte Proliferation Assay

Spleen from sacrificed mouse was removed aseptically into a Petri dish containing culture medium (complete RPMI-1640 containing 5% (v/v) fetal bovine serum (FBS), 300 *μ*g/mL L-glutamine, 100 IU/mL penicillin, and 100 *μ*g/mL streptomycin). Splenocytes were released from the spleen by gentle disruption of the splenic capsule. The splenocytes were gently teased out and collected in a tube and the splenocytes were recovered by centrifugation (1,200 rpm × 10 min at 4°C). The splenocytes were seeded into 96-well plates (Falcon 3075, Becton Dickinson, NJ, USA) at 5 × 10^3^ cells/well and cultured in the presence of 10 *μ*g/mL of pure TT (Calbiochem, Germany), 1 *μ*g/mL of Concanavalin A (Con A) (Sigma-Aldrich Inc., St. Louis Missouri, USA), or 1 *μ*g/mL lipopolysaccharide (LPS) (Sigma-Aldrich Inc., St. Louis Missouri, USA) for 72 hours at 37°C in a humidified, 5% CO_2_ incubator. Splenocyte proliferation was measured using the MTT assay according to the manufacturer's standard protocol (Roche Applied Science, Germany). The productions of cytokines by these cells were measured by ELISA.

### 2.5. Cytokine Analysis

After 72 hours, the supernatants from the splenocytes cultures were recovered by centrifugation (12,000 rpm × 10 min at 4°C). The amount of cytokines (IFN-*γ*, IL-4, and TNF-*α*) in the supernatants was determined using commercial mouse cytokine ELISA kits (eBioscience, San Diego, CA, USA). The amount of cytokine produced is expressed as pg/mL. The detection limit of the cytokine ELISA kits was 8 pg/mL. 

### 2.6. Extraction of Vitamin E from the Mice Adipose Tissue for HPLC Analysis

Approximately 0.5 g of mice adipose tissue was placed into a 15 mL centrifuge tube and homogenised with a mixture of hexane, ethanol, and 0.9% sodium chloride (at the ratio of 4 : 1 : 1) at 10000 rpm for five minutes or until the tissue was reduced to a liquid form using a tissue homogeniser. The homogenate was then centrifuged at 2000 rpm for 10 minutes. The lipid-containing supernatant phase was transferred to 5 mL vials and dried down under nitrogen gas. The sample obtained was resuspended just before use in an appropriate amount of hexane (500 *μ*L to 2 mL) for analysis by high performance liquid chromatography (HPLC). Analytical HPLC was performed using the LC-10AT HPLC system as previously described [16]. The HPLC system consisted of a Shimadzu Model RF-10AXL fluorescence spectrophotometer, a column chamber and Shimadzu Class VP data acquisition software as described previously [17]. The HPLC column used was the YMC A-012, 5 *μ*m, 150 mm × 6 mm silica column. The excitation wavelength and emission wavelength of the fluorescence detector were set at 295 and 325 nm, respectively. The mobile phase was hexane-isopropyl alcohol (99.5/0.5, v/v) with a flow rate of 2 mL/min. Sample injection volume was set at 10 *μ*L and a standard solution of mixture of pure isomers of vitamin E (*α*-T and *α*-, *δ*- and *γ*-T3) was also injected accordingly into the system. The peak areas of the components in the sample were compared with those of the standards and were used for quantitative calculation.

### 2.7. Statistical Analysis

Data are presented as the mean ± SD. In all experiments, all the samples were assessed individually. Statistical comparisons were performed using one-way ANOVA, followed by *post hoc* pair wise comparisons with 95% confidence interval (*P* < 0.05). 

## 3. Results

### 3.1. Production of Anti-TT Antibodies

The amount of anti-TT antibody produced after the first TT vaccination, that is, V1, was significantly (*P* < 0.05) higher in the vitamin E supplemented groups when compared to the control mice (Figure 3). There were no significant differences (*P* > 0.05) in the anti-TT levels in all three experimental groups after the primary immunisation. However, following booster TT vaccinations, the TRF and *δ*-T3 supplemented mice produced significantly (*P* < 0.05) higher anti-TT antibody compared to control or *α*-T supplemented mice (Figure 3). The mice supplemented with *δ*-T3 produced the highest amount of anti-TT antibodies, that is, *δ*-T3 > TRF > *α*-T > control. 

### 3.2. Splenocyte Proliferation of in Response to Mitogen or Antigen

There were no significant (*P* > 0.05) differences in the proliferation of splenocytes harvested from the mice in the different treatment groups (Figure 4). 

### 3.3. Production of IFN-*γ*, IL-4, and TNF-*α*

The amount of IFN-*γ* produced by the Con A or TT-stimulated splenocytes from the vitamin E supplemented mice was significantly (*P* < 0.05) higher than that from the control mice (Figure 5(a)). Although a similar result was obtained for IL-4 production (Figure 5(b)), the amount of IFN-*γ* produced was found to be very much higher. In contrast, the amount of TNF-*α* produced by the LPS-stimulated splenocytes from the vitamin E supplemented mice was found to be significantly (*P* < 0.05) lower than that from the control mice (Figure 5(c)).

### 3.4. Quantification of Vitamin E in Adipose Tissues

Although the adipose tissue obtained from the *α*-T supplemented mice had the highest amount of *α*-T (80 *μ*g/mL) stored in their adipose tissue (Figure 6), the tissue did not contain other isomers of vitamin E. Similarly, the adipose tissue from the *δ*-T3 contained mostly (120 *μ*g/mL) this isomer and some lower levels of *α*-T (Figure 6). The level of *α*-T in the adipose tissue of the *δ*-T3 fed animals was similar to that observed in the adipose tissue from the vehicle-fed mice. In contrast, all the vitamin E isomers analysed were detected in the adipose tissue from the TRF-supplemented mice (Figure 6).

## 4. Discussion

Vitamin E is a family of eight natural compounds, which are divided into two broad groups, namely, the tocopherols and tocotrienols. The *α*-T has the highest bioavailability and it is the standard that is generally used to compare all the other isomers of vitamin E [19, 20]. The immune enhancing effects of *α*-T, have been intensively studied in animal [8–11] and human models [7, 16, 17, 21]. There are some studies and only a few reports that describe the immunomodulatory effects of tocotrienols [11, 16, 17]. In this study, the effects of daily supplementation of three natural forms of vitamin E found in palm oil (*α*-T, *δ*-T3, or TRF) on immune response to the TT vaccine were compared using a murine model. At the time this study was conducted, only two pure homologues of vitamin E (*α*-T and *δ*-T3) were available in the pure form. We have previously reported that supplementation of TRF augmented immune response to TT vaccine in healthy young human volunteers [17]. Hence, in this study the TRF was also included in this study as a positive control. The TT vaccine was chosen as the antigen for this study as we wanted to link the findings from this study to what we had previously found in a human study that we had previously conducted using a similar model [17]. In addition, the TT vaccine is a well characterised and potent immunogen of bacterial origin, reported to induce long-lasting immune responses [22]. The ability to mount recall responses to TT is considered to be indicative of a healthy and intact immune system [23]. 

The results show that after the primary TT immunisation, the anti-TT titres obtained were significantly elevated in all the vitamin E supplemented groups compared to vehicle-fed animals. After the third TT vaccine, the anti-TT titres were significantly elevated in *δ*-T3 and TRF-fed animals compared to the *α*-T supplemented mice. However, the *α*-T fed mice produced significantly higher anti-TT when compared to the mice in the vehicle-fed group. These findings suggest that daily supplementation of *δ*-T3 or TRF has a more potent ability to augment secondary immune responses to specific antigens compared to *α*-T. We have previously demonstrated that TRF supplementation enhances the production of anti-TT antibodies of the IgG class and enhances the production of IFN-*γ* by Con A or TT-stimulated peripheral blood leucocytes [17]. The IFN-*γ* is the signature cytokine of TH1-immune responses, which include promotion of cell-mediated immune and classswitching to the IgG class of antibody [12]. The data suggest that supplementation with *δ*-T3 or TRF may be able to sustain the levels of IFN-*γ* in these animals and as such was able to produce significantly higher titres of anti-TT antibodies in the mice that were fed with these forms of vitamin E. Our results support a previous study that found supplementation of vitamin E can improve cell-mediated immunity [24]. Supplementation of vitamin E has also been reported to improve the decreased cellular immune functions caused by aging in mice [25] and rats [26]. However, in the present study, we found that supplementation with TRF or *δ*-T3 significantly enhanced the antigen-specific immune response and cytokine production in young, six-week-old BALB/c mice, which suggests supplementation with TRF or *δ*-T3 can also improve immune responses in younger mice. The differences in findings between our study and previous ones [25, 26] could be because in our study, we were able to measure antigen-specific responses whilst the previous studies did not involve any antigenic challenge. We have previously also shown that supplementation with TRF or alpha-tocopherol did not induce any significant immunomodulatory changes in healthy young adults [16]. 

There was a significant increase in the proliferation of Con A or TT-stimulated splenocytes harvested from the vitamin E supplemented groups as compared to control animals. However, within the vitamin E treated group, there were significant differences in the proliferation of the splenic lymphocytes. These findings suggest oral supplementation of vitamin E, regardless of whether it is tocopherol or tocotrienol, was efficacious in enhancing mitogen or specific antigen-induced proliferation of splenic lymphocytes. The T-helper (TH) cells are divided into two main types of cells with regard to their cytokine productivity, that is, TH1 cells which produce IFN-*γ* and IL-2 and TH2 cells which produce IL-4 and IL-5 [12, 26]. Splenocytes from the vitamin E supplemented mice that were cultured with Con A or TT produced significantly higher levels of IFN-*γ*. The amount of IFN-*γ* produced was significantly augmented after the third dose of the TT vaccine in all the three vitamin E treated groups as compared to the vehicle-fed animals. Within the vitamin E supplemented groups, animals fed with *δ*-T3 produced significantly higher levels of IFN-*γ* in Con A stimulated cultures as compared to the *α*-T, TRF, and vehicle-fed mice animals. The production of IL-4 following stimulation by TT was also significantly elevated in all the vitamin E treated groups as compared to vehicle-fed mice but the levels did not differ significantly amongst the vitamin E supplemented groups. These findings differ from a previous report that dietary tocopherol and tocotrienol supplementation only enhanced IFN-*γ* production by the mesenteric lymph node lymphocytes but not by the splenic lymphocytes [11]. However, it should be noted that in the previous study [11], the rats were not given any immunogenic challenge, so the authors may have only managed to measure nonspecific proliferation of splenic and mesenteric lymph node lymphocytes as well as IFN-*γ* production in their experimental animals. In contrast, in our study, the animals were fed with different forms of vitamin E and vaccinated thrice with the TT vaccine. So it is possible that the enhanced IFN-*γ* production by splenic lymphocytes in our study was due to the presence of the antigenic challenge. The production of IL-4 was found to be significantly higher in the vitamin E supplemented groups when compared to the vehicle group. However, the levels of IL-4 produced was found to be much lower than the IFN-*γ*. The IFN-*γ* is reported to be one of the signature cytokines for TH1-type immune response [27], our findings suggest that vitamin E supplementation may enhance cell-mediated immune response.

The LPS-stimulated splenic lymphocytes from the mice supplemented with different isomers of vitamin E were found to be significantly lower than those from the vehicle group. However, there were no significant differences observed between the vitamin E supplemented groups. This finding is in agreement with a previous report that showed long-term supplementation of vitamin E can suppress production of IL-6 and TNF-*α* [28]. Based on these findings, it is conceivable to surmise that vitamin E plays a pivotal role within the cytokine network, which contributes to the regulation of inflammatory and immune responses.

The concentrations of vitamin E isomers in the adipose tissue of the mice were analysed because vitamin E is a fat-soluble compound, which is stored in subcutaneous adipose tissue [29]. In addition, the concentrations of tocopherols and tocotrienols in adipose tissue may be a better indicator of its abundance than plasma levels over a relatively long time, because the former are generally not affected by rapid changes in the level of plasma lipoproteins or by acute changes in its intake [30–33]. The concentration of *δ*-T3 was significantly augmented in animals supplemented with *δ*-T3. This homologue was not detectable in the vehicle or the *α*-T fed animals. In the TRF-supplemented animals, we were able to detect most of the natural forms of vitamin E such as *α*-T, *α*-T3, *γ*-T3, and *δ*-T3. This is not surprising as TRF contains all these isomers, albeit varying concentrations. The *α*-T form was found to be present in the adipose tissues of animals in the vitamin E treated and vehicle groups. This was most likely due to the presence of *α*-T that might be present in the standard food pellets used to feed the mice. In the last two decades, studies on understanding how dietary vitamin E is transported to the tissues have focused primarily on the *α*-T [31, 32]. It has been shown that *α*-T binds to a transfer protein known as *α*-T transfer protein (TTP), which mediates the secretion of this vitamin into the plasma [31, 34]. As compared to tocotrienols, the *α*-T has a higher affinity to bind to TTP [30] and as such this led to the notion that availability of dietary T3 in tissues is negligible [32]. In rats fed with various isoforms of tocotrienols, it was shown that *α*-T3 had the highest oral bioavailability and lowest clearance rate whilst there were no significant differences between the *γ*- and *δ*-T3 [20]. Although in the study by Yap et al. [20], the authors did not include a group fed with *α*-T, there are other reports which have shown that *α*-T has a higher bioavailability and lower clearance rate when compared to tocotrienols [29, 30]. A recent study has shown that the postprandial metabolic fate of TRF is significantly different from that of *α*-T [34].

In conclusion, this study shows that daily supplementation of vitamin E can enhance immune response to a specific antigen. The highest immune response to the TT vaccine was observed in the *δ*-T3 supplemented mice, followed by TRF and *α*-T. In addition, vitamin E supplementation appears to favour a TH1 response and appears to inhibit production of TNF-*α* from LPS-stimulated murine splenocytes.

## Figures and Tables

**Figure 1:** Chemical structure of (a) alpha-tocopherol and (b) the main homologues of tocotrienols.

**Figure 2:** The study protocol. Mice in the experimental groups were fed with 1 mg of the vitamin E isomers (*α*-T, *δ*-T3, or TRF) from day 0 until the mice were sacrificed. Control mice were given 0.1 ml of the vehicle (Soya oil), which was used to make the various vitamin E preparations. All animals were vaccinated with tetanus toxoid vaccine on day 14 (TT first). Booster doses of the TT vaccine were given on days 28 (TT second) and 42 (TT third).

**Figure 3:** The mice in the various groups were fed with Soya oil (vehicle), alpha-tocopherol (alpha-T), delta-tocotrienol (delta-T3), or tocotrienol-rich fraction (TRF). Mice in all groups were immunised intramuscularly with 4 Lf/mL of TT on days 14, 28, and 42. Serum was collected on day 0 (PB), day 28 (V1) and day 56 (V2). Serum levels of anti-TT were determined by ELISA. The values are presented as mean ± standard deviation (S.D.). The *δ*-T3 supplemented mice produced the highest anti-TT titres following booster vaccination. [*significant (*P* < 0.05) difference from vehicle-fed group;  ^#^significant difference from *α*-T supplemented group].

**Figure 4:** The mice in all groups were sacrificed two week after the third TT vaccination (day 56). Splenocytes were aseptically removed from the mice and cultured in the presence of Concanavalin A (Con A), tetanus toxoid (TT), or lipopolysaccharide (LPS) at 37°C for 72 hours in a humidified 5% CO_2_ incubator. Proliferation of the splenocytes was measured by the MTT method. The values are presented as mean ± standard deviation (S.D.).

**Figure 5:** Production of (a) IFN-*γ* and (b) IL-4 by Con A or TT-stimulated splenocytes and (c) TNF-*α* from LPS-stimulated splenocytes harvested from mice fed with Soya oil (vehicle), *α*-tocopherol (alpha-T), *δ*-tocotrienol (delta-T3), or TRF. Sera from unmanipulated animals (naive) were used as baseline check. [*significant (*P* < 0.05) difference between the control and experimental groups].

**Figure 6:** Adipose tissue was obtained from mice fed with Soya oil (vehicle), *α*-tocopherol (alpha-T), *δ*-tocotrienol (delta-T3), or TRF and analysed using HPLC to determine concentrations of (a) total vitamin E and (b) *α*-T, and tocotrienol isomers in this tissue. [*significant (*P* < 0.05) differences between experimental and control groups].
